# Knockdown of miR-214 Alleviates Renal Interstitial Fibrosis by Targeting the Regulation of the PTEN/PI3K/AKT Signalling Pathway

**DOI:** 10.1155/2022/7553928

**Published:** 2022-10-15

**Authors:** DongHua Hou, Qi Wu, SiYu Wang, Shuo Pang, Hui Liang, HuiYan Lyu, Lu Zhou, Qiao Wang, Lirong Hao

**Affiliations:** ^1^Department of Nephropathy and Hemodialysis, First Affiliated Hospital of Harbin Medical University, Harbin, China; ^2^Department of Nephropathy, Southern University of Science and Technology Hospital, Shenzhen, China; ^3^Department of Nephrology, Tangdu Hospital, The Air Force Military Medical University, Xi'an, China; ^4^School of Chemistry and Chemical Engineering Harbin Institute of Technology, Harbin, China

## Abstract

The microRNA-214 (miR-214) precursor is formed by the DNM3 gene on human chromosome 1q24.3, which is encoded and transcribed in the nucleus and processed into mature miR-214 in the cytoplasm. Association of miR-214 with the interstitial fibrosis of the kidney has been reported in existing research. Renal interstitial fibrosis is considered necessary during the process of various renal injuries in chronic kidney disease (CKD). One of the important mechanisms is the TGF- (transforming growth factor-) *β*1-stimulated epithelial interstitial transformation (EMT). The specific mechanisms of miR-214-3p in renal interstitial fibrosis and whether it participates in EMT are worthy of further investigation. In this paper, we first demonstrated modulation of the downstream PI3K/AKT axis by miR-214-3p through targeting phosphatase and tension protein homologues (PTEN), indicating the miRNA's participation in unilateral ureteral obstruction (UUO) nephropathy and TGF-*β*1-induced EMT. We overexpressed or silenced miR-214-3p and PTEN for probing into the correlation of miR-214-3p with PTEN and the downstream PI3K/AKT signalling pathways. According to the results of the study, miR-214-3p overexpression silenced PTEN, activated the PI3K/AKT signalling pathway, and exacerbated EMT induced by TGF-*β*1, while miR-214-3p knockdown had the opposite effect. In miR-214-3p knockdown mice, the expression of PTEN was increased, the PI3K/AKT signalling pathway was inhibited, and fibrosis was alleviated. In conclusion, miR-214-3p regulates the EMT of renal tubular cells induced by TGF-*β*1 by targeting PTEN and regulating the PI3K/AKT signalling pathway. Furthermore, miR-214-3p knockdown can reduce renal interstitial fibrosis through the PTEN/PI3K/AKT pathway.

## 1. Introduction

In the course of CKD (chronic kidney disease) evolution, most kidney damage undergoes the same pathological stage, namely, renal interstitial fibrosis. The typical characteristics involve extracellular matrix (ECM) protein overproduction and deposition, including increased levels of collagen I (COL1) and fibronectin (FN) [1, 2]. Epithelial mesenchymal transformation (EMT) refers to transforming growth factor *β* (TGF*β*) driving the process by which renal tubular epithelial cells (TECs) acquire mesenchymal cell features after losing epithelial features. The EMT process in TECs exerts a pivotal function in the interstitial fibrosis of the kidney [3]. However, we lack an understanding of the underlying molecular mechanisms. Studies on the molecular mechanism of renal interstitial fibrosis can provide new possibilities for inhibiting fibrosis [4, 5].

miRNAs (microRNAs) refer to small 19–25 nucleotide-long molecules of noncoding RNAs that are highly conserved. By combining with the 3′UTR (3′-untranslated region) of the target posttranscriptional genes, the effect of regulating gene expression is realized [6]. miRNAs are associated with a variety of kidney diseases, especially fibrotic diseases, by regulating cell proliferation, apoptosis, differentiation, and development [7, 8]. miRNAs participate in various kidney diseases by regulating corresponding signalling pathways and cell activities [9]. For example, miR-107 induces TNF-*α* secretion by targeting bispecific phosphatase 7 (DUSP7) in endothelial cells, inducing renal tubular cell damage in septic AKI [10]; miR-21 inhibits the inflammatory response and apoptosis of renal tubular epithelial cells by stimulating the phosphatidylinositol 3-kinase (PI3K)/protein kinase B (AKT) pathway, improves AKI induced by I/R [11], and inhibits apoptosis of AKI renal cells induced by sepsis through the PI3K/AKT signalling pathway [12].

miR-214-3p is a microRNA encoded by the DNM3 gene in the q24.3 region of chromosome 1, which is highly conserved in vertebrates [13]. In the nucleus, pri-miR-214-3p is produced by transcription initiated by RNA polymerase II or III. Subsequently, the precursor miR-214-3p is formed from pri-miR-214-3p due to the action of endonuclease Drosha and its cofactor [14–16]. The precursor miR-214-3p is transported to the cytoplasm and processed by the endonuclease Dicer to gradually form mature miR-214-3p [17–19]. miR-214-3p exists in multiple organs and is involved in different kidney diseases (Human miRNA Expression Database). For example, previous research demonstrated prominent miR-214-3p overexpression in the kidney injury models and was associated with the development of fibrosis [9, 20]. miR-214-3p has been confirmed to increase expression in renal interstitial fibrosis in vivo, and this change does not depend on the TGF-*β* pathway [9, 20]. miR-214-3p antagonism can be regarded as a new treatment for renal tubulointerstitial fibrosis [9, 20]. Therefore, the specific mechanism of miR-214-3p in renal tubulointerstitial fibrosis needs further study.

There is increasing evidence that phosphatase and tensin homologue (PTEN) is a negative fibrosis regulator in diverse organs, including the lungs, heart, and liver [21–23]. PTEN can reduce the activity of the PI3K (phosphatidylinositol 3-kinase)/AKT (protein kinase B) axis. PTEN inhibits the effect of this pathway on cells and is an endogenous negative regulator [24–26]. The PI3K/AKT axis initiation is linked to the pathogenesis of various tumours [27] and is an important mediator related to organ fibrosis [28–30]. Accumulating evidence shows that PTEN in kidney cells can be targeted and regulated by miRNAs, which in turn affects AKT activation [31]. Flufenidone suppresses the functionality of nicotinamide adenine dinucleotide phosphate oxidase during renal interstitial fibrosis by relying on the PI3K/AKT axis [30]. These studies confirm that the EMT process of renal tubulointerstitial fibrosis is related to PTEN/PI3K/AKT. In a diabetic environment, low miR-214-3p expression leads to PTEN overexpression by targeting PTEN, thus improving renal glomerular hypertrophy [32, 33]. However, there are few studies on the mechanism of miR-214-3p during renal interstitial fibrosis.

The above studies confirm the relationship between the loss of PTEN in the renal interstitium and renal interstitial fibrosis. The increased expression of miR-214-3p can promote EMT of renal tubular epithelial cells and renal interstitial fibrosis. Previous research and miRNA databases have shown that miR-214-3p targets PTEN directly [32–34]. Therefore, we assume that miR-214-3p regulates the PI3K/AKT signalling pathway through targeting PTEN and promotes EMT and renal interstitial fibrosis. Intervening with the expression of miR-214-3p and PTEN may be a new method to alleviate renal fibrosis. Thus, we first used the unilateral ureteral obstruction (UUO) mouse model and human tubuloepithelial (HK-2) to study the relationship between miR-214-3p and PTEN in renal interstitial fibrosis. We demonstrate that miR-214-3p reduces PTEN levels by binding to the 3′-UTR of PTEN mRNA, thereby acting on the PI3K/AKT signalling pathway to reduce the EMT of renal tubular cells triggered by TGF-*β*1. Knockdown of miR-214-3p can relieve renal interstitial fibrosis through the PTEN/PI3K/AKT pathway.

## 2. Materials and Methods

### 2.1. Cell Culture and Transfection

We chose DMEM/F12 (Gibco, USA) as the human tubuloepithelial cell (HK-2) culture medium. The medium was supplemented with 1% penicillin, 1% streptomycin, and 10% foetal bovine serum (Gibco, USA) according to the ratio. The cells were placed in a humidified incubator (5% CO_2_, 37°C). HK-2 cells at a confluency of 50-60% were placed in a 24-well plate and starved for 48 h (0.2% foetal bovine serum) (Biological Industries, Israel). After starvation, the medium was changed, and 10 ng/mL TGF-*β*1 (Solarbio, China) was added to the culture medium for 48 h. Then, LV-miR-214-OE (a lentivirus expressing the sequence of human pri-miR-214-3p), LV-miR-214-KD (a lentivirus having an oligonucleotide against the mature sequence of human miR-214-3p), or LV-NC-OE/LV-NC-KD negative controls were transfected into HK-2 cells for 12 h. The medium containing the lentivirus was replaced with fresh medium. The lentivirus used was from Wanlei Biological Technology (Shenyang, China).

### 2.2. Transient Transfection

To investigate the role of PTEN, we chose Lipofectamine 2000 (Invitrogen, USA) for transient transfection of TGF-*β*1-stimulated logarithmic HK-2 cells with 50 nM si PTEN (PTEN siRNA) and scr-siRNA (scrambled siRNA; both from GenePharma, China) for a duration of 8 h. The same method was used to transfect pcDNA3.1-PTEN overexpression plasmids (including human PTEN cDNA, PTEN-OE plasmid, Gene, China) or blank control pcDNA3.1 plasmid (BC plasmid, Gene, China) in LV-miR-214-OE or LV-NC-OE cells for 8 h.

### 2.3. Immunofluorescence Analysis

Each group of cells was spread on sterile coverslips, subsequently immobilized in paraformaldehyde (4%) and, 25 min later, washed away. A 5 min infiltration of the cells proceeded using Triton X-100 (0.15%) at ambient temperature, followed by a 1 h blockage using goat serum (10%; Beyotime, China) for 1 h. Primary antibody (anti-PTEN, 1 : 50 dilution, Wanlei; anti-PI3K 1 : 200 dilution, Abcam) was incubated overnight at 4°C. At 37°C, the cells were incubated with secondary antibody (Cy3-labeled goat anti-rabbit IgG, 1 : 500 dilution, Proteintech) for 1 h after overnight incubation. Finally, a 5 min staining of the cellular nuclei was accomplished using DAPI (Solarbio, China). For the image assessment, the Eclipse Ti-s microscopes (Nikon) adopting constant exposure were utilized. The statistical analysis of fluorescence intensity was accomplished via the Image-Pro Plus 6.0 (Media Cybernetics).

### 2.4. UUO Model

The experimental animals came from the Harbin Medical University's Laboratory Animal Center. The experimental protocol was approved by the Ethics Committee on the Laboratory Animal Use and Welfare of the First Hospital Affiliated to Harbin Medical University in China's Harbin. We selected wild-type male C57BL/6 mice for experiments and obtained mice from specific pathogen-free (SPF) conditions. The mice were 8 weeks old and weighed 20-25 g. The experimental mice were randomized into 4 groups, with 6 mice per group. In addition to a sham operation group, the other three groups were UUO groups. The UUO group was anaesthetized with pentobarbital sodium (40 mg/kg, IP), and 4-0 silk ligate was used to ligate the left ureter. In the sham group, the mice were treated in a similar way but did not undergo ureteral ligation. Mice were sacrificed 14 days after UUO to collect obstructed kidneys for real-time PCR, Western blotting, histology, and immunohistochemistry.

### 2.5. Virus Injection

C57BL/6 mice had ad libitum access to food and water and were kept under conventional experimental conditions (light and dark cycle for 12 h; 22-24°C). Two groups of UUO mice were injected with 100 *μ*L of lentivirus (LV-miR-214-KD) (1 × 10^9^ TU/mL) and 100 *μ*L of control lentivirus (LV-NC-KD) (1 × 10^9^ TU/mL) via the tail vein 7 and 14 days before the operation. On the 14th day after UUO, half of the left kidney of the sacrificed mice was fixed in 10% formalin. After tissue dehydration, paraffin embedding, and sectioning, histological and immunohistochemical analyses were carried out.

### 2.6. Renal Immunohistochemistry and Histopathology

To evaluate histological changes in the kidney, such as interstitial fibrosis, paraffin sections of renal tissue (3 *μ*m) were subjected to haematoxylin-eosin (HE) and Masson's trichrome staining. We detected collagen fibre deposition by a Masson staining kit (Baso, China). The blue–purple collagen deposition area indicated the severity of interstitial fibrosis. We deparaffinized renal sections, hydrated them, and rinsed them with distilled water. A 25 min treatment proceeded with 3% hydrogen peroxide (H_2_O_2_) at ambient temperature. Following a 30 min blockage using goat serum (10%; Solarbio, China), the cells were bound to primary antibodies (anti-PTEN, 1 : 200 dilution, Wanlei; anti-PI3K, 1 : 600 dilution, Absin) overnight at 4°C. After overnight incubation, the sections were subjected to a 1 h incubation using a 1 : 500 diluent of peroxidase-labeled secondary antibody (Jackson ImmunoResearch) under a 37°C condition. Then, we developed immunohistochemically stained tissue sections with DAB for 30 min and counterstained them with haematoxylin. Two blinded researchers independently observed all slides and chose five fields of view in a random manner from every section. The percentage of positively stained areas was estimated via the Image-Pro Plus 6.0.

### 2.7. Western Blot Analysis

Cell and tissue proteins were extracted with a RIPA extraction kit (Wanlei, China). A 10% SDS–PAGE gel was used to isolate the same amount of protein (50 *μ*g). The proteins were transferred to a PVDF membrane (Roche, USA). At room temperature, a 2 h sealing was accomplished using nonfat milk (5%). At 4°C, the primary antibodies were incubated overnight, including anti-PTEN (1 : 1000 dilution, Proteintech), anti-PI3K (1 : 1000 dilution, Abmart), anti-p-AKT (1 : 1000 dilution, Abmart), anti-AKT (1 : 2000 dilution, Abmart), anti-*α*-SMA (1 : 1000 dilution, Wanlei), anti-COL1 (1 : 500 Wanlei), anti-FN (1 : 1000 dilution, Wanlei), and anti-GAPDH (1 : 3000 dilution, Abmart) antibodies. The membranes were nurtured for 1 h using horseradish peroxidase (Wanlei, China) under ambient temperature. The protein bands were detected via an advanced ECL kit (Beyotime, China).

### 2.8. Real-Time PCR

The membranes were nurtured for 1 h using horseradish peroxidase (Wanlei, China) under ambient temperature. The protein bands were detected via an advanced ECL kit (Beyotime, China). Reverse transcription of the overall RNA as template cDNA proceeded through PrimeScriptTM RT Master Mix (TOYOBO, Japan) for mRNA. The qRT-PCR amplification was assessed with a real-time PCR system from Applied Biosystems. All amplifications were repeated three times. We used the comparative Ct (2-*ΔΔ*Ct) method to measure the related gene levels. The internal reference genes were GAPDH and U6. According to the primer design principle, primers were designed by Primer 5.0 operation software. Three sets of forward and reverse primers were designed for each target gene primer, which were synthesized by Generay Biotechnology Company (China). The appropriate primers of the target gene were selected by pre-experiments (Table 1).

### 2.9. Determination of Dual-Luciferase Reporter Activity

When the HK-2 cells were in the log phase, we used Lipofectamine 2000 (Invitrogen, USA) to cotransfect mimics of miR-214-3p or NC plus MUT (mutant) or WT (wild-type) PTEN 3′-UTR. The HK-2 cells treated with different transfections after 48 h were subjected to the luciferase potential assessment through the dual-luciferase reporter assay (Abcam, UK).

### 2.10. Statistical Analysis

We used GraphPad Prism 7.0 to perform statistical analysis on the experimental data. The data represent three independent repeated experiments, rendered as the means ± SDs (standard deviations). Student's *t* test was employed to make the pairwise comparisons, while univariate ANOVA was adopted for comparisons among 3 or more groups. And then, Tukey's multiple comparison post hoc test was applied. Usually, differences were regarded as significant with the *P* values being less than 0.05.

## 3. Results

### 3.1. miR-214-3p Expression Increased and PTEN Expression Decreased

For the exploration of the miR-214-3p and PTEN levels, we selected HK-2 cells and C57BL/6 mice as the research objects. The results revealed that HK-2 cells exhibited typical mesenchymal cell morphology after 48 h of TGF-*β*1 treatment, and the morphology changed significantly in contrast to the control (Figure 1(a)), implying the EMT elicitation by TGF-*β*1 in the HK-2 cells based on cell morphology. The UUO model is a commonly used experimental model of renal interstitial fibrosis. We established the UUO mouse model by obstructing its left renal ureter and performed histochemical staining to observe renal pathological changes. Compared with the sham group, HE and Masson staining revealed that UUO mice showed the following typical characteristics: inflammatory cell infiltration, tubular dilatation, and interstitial fibrosis (Figure 1(b)), indicating that the UUO group developed renal interstitial fibrosis. The miR-214-3p, PTEN, COL1, FN, and *α*-SMA expressions were examined through qRT–PCR analysis, showing that the level of miR-214-3p in HK-2 cells stimulated with TGF-*β*1 was greatly upregulated in relative to the control (Figure 1(c)). The miR-214-3p level in the fibrosis group (UUO) was also significantly increased in the in vivo experiment (Figure 1(d)). Additionally, the mRNA level of PTEN was downregulated, and fibrosis-related mRNA levels, such as *α*-SMA, COL1, and FN, were upregulated in HK-2 cells after stimulation with TGF-*β*1 and in UUO mice (Figures 1(e) and 1(f)). The Western blot results also confirmed this finding (Figures 1(g)–1(j)).

### 3.2. miR-214-3p Targeted PTEN

According to Figure 2(a), binding of miR-214-3p to the PTEN mRNA's 3′UTR was validated according to the TargetScan and miRanda, two bioinformatics software. Transfection of HK-2 cells was accomplished using mimics of miR-214-3p and NC. The miR-214-3p expression was upregulated greatly after 48 hours for the miR-214-3p group (Figure 2(b)). Based on the dual-luciferase reporter assay outcomes, when HK-2 cells were cotransfected using miR-214-3p/NC mimics plus WT/Mut PTEN 3′-UTR, the luciferase activity of the WT PTEN 3′-UTR decreased by the mimic of miR-214-3p, while did not in the case of the Mut PTEN 3′-UTR (Figure 2(c)). Furthermore, Western blot results showed that miR-214-3p greatly reduced PTEN expression in either the TGF-*β*1 treatment group or the negative control group (Figure 2(d)).

### 3.3. miR-214-3p Regulates EMT of HK-2 Cells Triggered by TGF-*β*1 by Targeting PTEN/PI3K/AKT

To probe deeper into the miR-214-3p's specific mechanisms in the EMT event of TGF-*β*1-processed HK-2 cells, LV-miR-214-KD, LV-miR-214-OE, LV-NC-KD, or LV-NC-OE were used for cellular transfection. As revealed by the results, miR-214-3p was obviously enhanced for the LV-miR-214-OE group, while notably decreased for the LV-miR-214-KD group (Figure 3(a)). miR-214-3p upregulation led to elevated levels of fibrosis biomarkers, including *α*-SMA, COL1, and FN, while its silencing resulted in declines of these levels, suggesting its role in adjusting the EMT of HK-2 cells triggered by TGF-*β*1 (Figures 3(c), 3(d) and 3(f)). Upregulating miR-214-3p reduced PTEN levels but increased PI3K and p-AKT levels (Figures 3(b), 3(d), and 3(e)). Silencing miR-214-3p upregulated PTEN levels but decreased PI3K and p-AKT levels (Figures 3(b), 3(d), and 3(e)). qRT–PCR and Western blot methods confirmed that miR-214-3p regulated the PTEN/PI3K/AKT pathway (Figures 3(b)–3(f)). Furthermore, immunofluorescence staining of PTEN and PI3K revealed the same results (Figures 3(g)–3(j)). This experiment confirmed that miR-214-3p mediated EMT induced by TGF-*β*1 via the PTEN/PI3K/AKT pathway.

### 3.4. PTEN Downregulation Activated the PI3K/AKT Signalling Pathway, Leading to TGF-*β*1-Induced EMT

In order to show the function of PTEN in TGF-*β*1-induced EMT, transfection of HK-2 cells was accomplished using si-PTEN and scr-siRNA after 48 hours of TGF-*β*1 treatment. PTEN expression in the si-PTEN group was greatly reduced, accompanied by upregulated synthesis of *α*-SMA, COL1, and FN and upregulated activity of the PI3K/AKT pathway proteins (Figures 4(a) – 4(e)). As validated by qRT–PCR plus WB, PTEN downregulation enhanced the levels of fibrosis-related indicators and PI3K/AKT pathways in TGF-*β*1-induced EMT (Figures 4(a)–4(e)). Immunofluorescence staining of PTEN and PI3K also confirmed these trends (Figures 4(f)–4(h)). These findings indicated that PTEN downregulation could promote the TGF-*β*1-triggered EMT through the PI3K/AKT axis initiation.

### 3.5. PTEN Was Essential for PI3K/AKT Pathway Activation and TGF-*β*1-Induced EMT in miR-214-3p-Overexpressing Cells

To further confirm that PI3K/AKT pathway activation and EMT of HK-2 cells caused by miR-214-3p overexpression were achieved through PTEN downregulation, EMT cells stimulated by TGF-*β*1 were divided into four groups and cotransfected with LV − NC − OE + BC, LV − NC − OE + PTEN OE, LV − miR − 214 − OE + BC, and LV − miR − 214 − OE + PTEN OE. PTEN expression was lower, the PI3K/AKT pathway was overactivated, and the levels of fibrosis markers were upregulated in the LV − miR − 214 − OE + BC group (Figures 5(a) – 5(e)). However, the overexpression of PTEN in the LV − miR − 214 − OE + PTEN − OE group significantly eliminated the abovementioned abnormal changes caused by miR-214-3p overexpression (Figures 5(a)–5(e)). Immunofluorescence analysis showed the same results (Figures 5(f)–5(h)). These data illustrated that miR-214-3p activates the PI3K/AKT signalling pathway and TGF-*β*1-induced EMT mainly through a PTEN-dependent mechanism.

### 3.6. Knockdown of miR-214-3p Reduced Renal Interstitial Fibrosis through the PTEN/PI3K/AKT Pathway

Finally, we used animal experiments to explore whether knockdown of miR-214-3p could relieve renal interstitial fibrosis and was linked to the PTEN/PI3K/AKT axis. LV-miR-214-KD and LV-NC-KD were injected via the tail vein into UUO mice. Compared with the UUO group, the LV-miR-214-KD group exhibited significantly decreased expression of miR-214-3p (Figure 6(a)). In accordance with the results of HE and Masson staining, we found that compared with UUO mice, UUO mice with miR-214-3p knockdown had significantly reduced interstitial fibrosis (Figure 6(b)). In UUO mice with miR-214-3p knockdown, reduced collagen deposition and low expression of fibrosis-related markers (*α*-SMA, COL1 and FN) were observed (Figures 6(c), 6(e), 6(f), and 6(h)). Furthermore, PTEN expression increased and PI3K and p-AKT levels decreased after treatment using the miR-214-3p inhibitor, and these results were the same as in the in vitro experiments (Figures 6(d), 6(f), and 6(g)). PTEN and PI3K were found mainly in renal tubular cells of the renal interstitium according to immunohistochemistry. The kidney PTEN level of UUO mice declined in contrast to that in the sham mice; however, silencing miR-214-3p reversed this change, and the PTEN level increased (Figures 6(i) and 6(j)). PI3K expression was opposite to that of PTEN (Figures 6(k) and 6(l)). This indicated that knockdown of miR-214-3p reduced renal fibrosis by overexpressing PTEN and inhibiting the PI3K/AKT pathway.

## 4. Discussion

Many studies on kidney-related diseases, such as diabetic nephropathy and acute kidney injury models, have revealed the role of miR-214 [9, 35, 36], but the mechanism of miR-214 in renal interstitial fibrosis has rarely been investigated. According to our research, we confirmed that miR-214-3p levels were upregulated, PTEN expression was decreased in UUO mice, and this effect was related to renal interstitial fibrosis (Figure 1), which was consistent with existing reports [20, 37]. We found that the expression of miR-214 and PTEN during the EMT process of HK2 cells induced by TGF-*β*1 was the same as that observed in vivo (Figure 1). Through online prediction software analysis and dual luciferase experiments, miR-214-3p was confirmed to target PTEN (Figure 2). We found that after si-PTEN silencing of PTEN, the PI3K/AKT axis was initiated, and the levels of fibrosis-related indicators increased. The level of PTEN was linked to the PI3K/AKT axis activity, as well as the TGF-*β*1-elicited EMT in HK-2 cells (Figure 4), suggesting that PTEN downregulation could promote EMT induced by TGF-*β*1 through activating the PI3K/AKT pathway. In terms of the exogenous modulation of the miR-214-3p level, treatment of these models with LV-miR-214-KD and LV-miR-214-OE was utilized, and its role in TGF-*β*-induced EMT was further studied. miR-214-3p upregulation intensified TGF-*β*-induced EMT, and silencing miR-214-3p had completely different effects (Figure 3). Combining the changes in PTEN and PI3K/AKT, we proved miR-214-3p's function in the EMT stimulated by TGF-*β*1, and this effect was achieved through the PTEN/PI3K/AKT pathway. By increasing the levels of PTEN and miR-214-3p, we demonstrated that the recovery of PTEN expression significantly eliminated the increase in PI3K/AKT pathway protein expression and fibrosis indicator upregulation resulted from the overexpression of miR-214-3p (Figure 5). This result suggested that PTEN was necessary for the EMT process induced by the miR-214-3p expression elevation. Finally, we verified through animal experiments that the miR-214-3p knockdown mitigated the interstitial fibrosis of the kidney through the PTEN/PI3K/AKT axis targeting (Figure 6).

PTEN is considered to be a tumour suppressor gene and has also been confirmed to have antifibrotic effects. Studies have confirmed that PTEN is related to glomerular hypertrophy in diabetic nephropathy [32, 33, 38–40] and can negatively regulate PI3K/AKT signalling activity [14]. Although there have been reports that PTEN and its regulation of PI3K/AKT activity play a role in various kidney diseases [41–43], the specific effect of the miR-214-3p/PTEN/PI3K/AKT axis on renal interstitial fibrosis remains to be explored and verified. In this article, miR-214-3p targeting of PTEN affected the downstream PI3K/AKT pathway, thereby regulating renal interstitial fibrosis and TGF *β*-induced EMT (Figure 4). miR-214 was proven to upregulate the PI3K/AKT pathway by targeting PTEN, thereby protecting cells from damage induced by hypoxia/reoxygenation (H/R) and reducing myocardial damage induced by ischaemia/reperfusion (I/R) and cardiomyocyte apoptosis [44, 45]. According to the results of this experiment, there may be a feedback regulatory loop between PTEN and PI3K/AKT in renal fibrosis induced by miR-214, but this conclusion needs further experimental confirmation.

miR-214 is abnormally expressed in tumours of many organs, including nasopharyngeal, pulmonary, hepatic, colorectal, pancreatic, cervical, and vesical carcinomas [46–48]. The pathogenesis and metastasis of these tumours are closely associated with the expression of miR-214 [49–52]. Knockdown of miR-214 was involved in the increase in apoptosis and fibrosis induced by cardiac I/R injury [44]. Previous studies and our research confirmed that miR-214 knockdown has a protective effect on the apoptosis of renal tubular epithelial cells, as well as the fibrosis of the kidney [20] (Figure 6). This result does not explain the specific mechanism in previous studies. TGF-*β* and downstream Smad signalling are generally considered to be the main signalling pathways in the process of fibrosis [53]. However, in the improvements in fibrosis after UUO induced by blocking the expression of miR-214 through gene knockout or drug inhibition, it has been confirmed that the regulation of miR-21 and miR-214 was independent of typical TGF-*β* signalling and the improvements in fibrosis [20]. In our study, we concluded that through the PTEN/PI3K/AKT axis targeting, the anti-miR-214 reduced TGF-*β*1-induced tubuloepithelial interstitial transformation and renal interstitial fibrosis. Studies have found that there are some non-Smad-mediated pathways of TGF-*β* for the TGF-*β*-elicited EMT in human pulmonary carcinoma cells, renal TECs, and renal sarcoma cells, and the PI3K/AKT pathway is a very important pathway [54]. Our conclusion was consistent with the existing research.

There are still some shortcomings in this research. The miR-214 downregulation was noted in the kidney following the miR-214 inhibitor administration intravenously, so the kidney may be the target organ of miRNA therapy. However, we did not explore the level of miR-214 in other tissues or organs, such as the liver, pancreas, and heart. These organs and tissues may have potential targets that are regulated by miR-214, which needs further research and verification. The study did not further explore the relationship between the classical pathway (TGF-*β*/Smad pathway) of renal interstitial fibrosis and the regulatory pathway of miR-214/PTEN/PI3K/AKT. Furthermore, we did not measure the expression of miR-214 and PTEN in human tissues, which would be needed to better determine expression changes in renal interstitial fibrosis from the three levels of cells, animals, and humans.

The results in Figure 1 of this study show the changes in miR-214-3p and PTEN in cell and animal renal fibrosis models, and Figure 2 verified the targeting relationship between miR-214-3p and PTEN. Based on these results, we further explored the changes in the PI3K/AKT signalling pathway and fibrosis during the changes in upstream miR-214-3p and downstream PTEN in Figures 3 and 4 to explore their internal regulatory relationship. Figure 5 shows that PTEN was a necessary factor for miR-214-3p to regulate the PI3K/AKT signalling pathway and fibrosis. Finally, the results in Figure 6 are from in vivo experiments to confirm the above results.

This study first confirmed that silencing miR-214 could alleviate renal interstitial fibrosis. miR-214-3p targeted PTEN to regulate the PI3K/AKT signalling pathway and participated in regulating the regulation of renal interstitial fibrosis. This research provides a new theoretical basis for exploring the role of renal tubular epithelial cells in renal interstitial fibrosis and a new target for treating TGF-*β*-induced renal interstitial fibrosis. Targeted intervention of renal miR-214-3p and PTEN will be of great significance for the clinical treatment of renal fibrosis.

## 5. Conclusions

In summary, this research shows that knockdown of miR-214-3p can reduce TGF-*β*1-induced tubulointerstitial interstitial transformation and renal interstitial fibrosis by upregulating PTEN and inhibiting the PI3K/AKT signalling pathway. Inhibiting miR-214-3p expression may offer a new therapeutic approach to inhibit renal interstitial fibrosis.

## Figures and Tables

**Figure 1:** miR-214-3p levels increased and PTEN levels decreased in vitro and in vivo. (a) HK-2 cells displayed typical mesenchymal morphology after TGF-*β*1 treatment for 48 h. Scale bars, 200 *μ*m. (b) Histopathological changes were observed by staining with Masson plus HE. Typical micrographs for various groups are displayed in the figure. Blue–purple collagen was deposited on the Masson-stained image. Scale bars, 100 *μ*m. (c, d) qRT–PCR-based expressions of miR-214-3p in the control, TGF-*β*1, sham, and UUO groups, and the internal reference miRNA was U6. (e, f) qRT–PCR-based mRNA expressions of PTEN, COL1, FN, and *α*-SMA. We chose GAPDH as an internal control for other genes. (g–j) Western blot results including PTEN, *α*-SMA, COL1, and FN in the control, TGF-*β*1, sham, and UUO groups. GAPDH was used as an internal reference for the other proteins. The data rendered are in terms of means ± SDs. *n* = 3. ^∗^*P* < 0.05, ^∗∗^*P* < 0.01, ^∗∗∗^*P* < 0.001, and ^∗∗∗∗^*P* < 0.0001 against the sham/control group.

**Figure 2:** miR-214-3p directly targeted PTEN. (a) The 3′-UTR of the human (hsa) and mouse (mmu) PTEN genes contained the miR-214-3p binding domain. (b) qPCR outcomes for the transfection efficiency of miR-214-3p mimics after 48 h transfection of the HK-2 cells. (c) The dual luciferase reporter analysis results after cotransfection of HK-2 cells using miR-214-3p/NC mimics plus WT/Mut PTEN 3′-UTR. The data rendered are in terms of means ± SDs, *n* = 3, ^∗∗∗^*P* < 0.001. (d) Western blotting detected PTEN levels after 48 h transfection of the TGF-*β*1 and control groups separately using mimic of miR-214-3p or NC. GAPDH served as an internal reference.

**Figure 3:** miR-214-3p regulated EMT via PTEN/PI3K/AKT. (a) miR-214-3p levels by qRT–PCR in control, TGF-*β*1, TGF − *β*1 + LV − miR − 214 − OE, TGF − *β*1 + LV − NC − OE, TGF − *β*1 + LV − miR − 214 − KD, and TGF − *β*1 + LV − NC − KD cells, and the internal reference miRNA was U6. (b, c) qRT–PCR-based expression outcomes for PTEN, PI3K, AKT, *α*-SMA, COL1, and FN at the mRNA level. (d–f) WB-based protein level outcomes for PTEN, PI3K, COL1, p-AKT, t-AKT, FN, and *α*-SMA in the control group, as well as in the TGF-*β*1, TGF − *β*1 + LV − miR − 214 − OE, TGF − *β*1 + LV − miR − 214 − KD, TGF − *β*1 + LV − NC − OE, and TGF − *β*1 + LV − NC − KD groups. In the result analysis, t-AKT and GAPDH served separately as the internal references for p-AKT and other proteins. (g, i) Typical immunofluorescence images showing PTEN and PI3K. PTEN was clearly distributed in the nucleus and cytoplasm. PI3K was mostly expressed in the cytoplasm. DAPI, blue; PTEN and PI3K, red; scale bars, 50 *μ*m. (h, j) Fluorescence intensity outcomes for the PTEN and PI3K. The data represented are in terms of means ± SDs, *n* = 3. ^∗^*P* < 0.05, ^∗∗^*P* < 0.01, ^∗∗∗^*P* < 0.001, and ^∗∗∗∗^*P* < 0.0001 against the TGF-*β*1/control group.

**Figure 4:** PTEN downregulation promoted EMT via the PI3K/AKT pathway. si-PTEN or scr-siRNA was transfected into HK-2 cells stimulated with TGF-*β*1. (a, b) qRT–PCR was performed to measure the mRNA levels of PTEN, PI3K, AKT, *α*-SMA, COL1, and FN in the control, TGF-*β*1, TGF − *β*1 + scr siRNA, and TGF − *β*1 + si − PTEN groups. (c–e) WB-based outcomes for the PTEN, PI3K, COL1, p-AKT, t-AKT, *α*-SMA, and FN levels. In the results analysis, t-AKT and GAPDH served separately as the internal references for p-AKT as well as other proteins. (f, h) Typical immunofluorescence images showing PTEN and PI3K. PTEN was clearly distributed in the nucleus and cytoplasm. PI3K was mostly expressed in the cytoplasm. DAPI, blue; PTEN and PI3K, red; scale bars, 50 *μ*m. (g, i) Fluorescence intensity of PTEN and PI3K. The data are rendered in terms of means ± SDs, *n* = 3. ^∗^*P* < 0.05, ^∗∗^*P* < 0.01, ^∗∗∗^*P* < 0.001, and ^∗∗∗∗^*P* < 0.0001 against the TGF-*β*1/control group.

**Figure 5:** Low PTEN expression was essential for miR-214-3p-overexpressing cells to enhance the PI3K/AKT pathway and EMT. HK-2 cells were divided into four groups after 48 h of TGF-*β*1 treatment and cotransfected with LV − NC − OE + BC, LV − NC − OE + PTEN OE, LV − miR − 214 − OE + BC, and LV − miR − 214 − OE + PTEN OE. (a, b) qRT–PCR outcomes for the PTEN, PI3K, AKT, COL1, FN, and *α*-SMA expressions at the mRNA level in the four groups. (c–e) WB expression outcomes for the PTEN, PI3K, COL1, p-AKT, t-AKT, *α*-SMA, and FN. In the results analysis, t-AKT and GAPDH served separately as the internal references for p-AKT and other proteins. (f, h) Typical immunofluorescence images showing PTEN and PI3K. PTEN was clearly distributed in the nucleus and cytoplasm. PI3K was mostly expressed in the cytoplasm. DAPI, blue; PTEN and PI3K, red; scale bars, 50 *μ*m. (g, i) Fluorescence intensity of PTEN and PI3K. The data are represented in terms of means ± SDs, *n* = 3. ^∗^*P* < 0.05, ^∗∗^*P* < 0.01, ^∗∗∗^*P* < 0.001, and ^∗∗∗∗^*P* < 0.0001 against LV − miR − 214 − OE + BC or LV − NC − OE + BC group.

**Figure 6:** Among the UUO mice, miR-214-3p downregulation alleviated renal interstitial fibrosis via the PTEN/PI3K/AKT axis. (a) qRT–PCR outcomes for the miR-214-3p expressions in the UUO, sham, UUO + LV − NC − KD and UUO + LV − miR − 214 − KD groups, and the internal reference miRNA was U6. (b) Histopathological changes were observed by Masson staining and HE staining. Typical images of each group are shown in the figure. Blue–purple collagen was deposited on the Masson-stained image. Scale bars, 100 *μ*m. (c) Statistical Masson staining results were expressed by semiquantitative analysis of the collagen deposition area. (d, e) qRT–PCR outcomes for the mRNA expressions of PTEN, COL1, FN, and *α*-SMA. For other genes, the internal reference used was GAPDH. (d–f) Western blot results of PTEN, PI3K, p-AKT, t-AKT *α*-SMA, COL1, and FN protein levels in all groups. In the results analysis, t-AKT and GAPDH served separately as the internal references for p-AKT and other proteins. (i, k) Typical immunohistochemical images of PTEN and PI3K. Scale bars, 100 *μ*m. (j, l) The levels of PTEN and PI3K were expressed by semiquantitative analysis of the positive staining area. Data are rendered in terms of means ± SDs. ^∗^*P* < 0.05, ^∗∗^*P* < 0.01, ^∗∗∗^*P* < 0.001, and ^∗∗∗∗^*P* < 0.0001 against the UUO/control group.

**Table 1:** qRT–PCR primers.

Gene	Primers (5′ to 3′)
Mmu and hsa miR-214-3p	F: ACAGCAGGCACAGACAGGCAG R: GTGCAGGGTCCGAGGTATTC
Mmu and hsa U6	F: GGAACGATACAGAGAAGATTAGC R: TGGAACGCTTCACGAATTTGCG
Mmu PTEN	F: CCCACCACAGCTAGAACTTATC R: CGTCCCTTTCCAGCTTTACA
Mmu PI3K	F: AAGGAGCTGGTGCTACATTATC R: CGCCTCTGTTGTGCATATACT
Mmu AKT	F: ACGACGTAGCCATTGTGAAG R: GCCGTTCCTTGTAGCCAATA
Mmu *α*-SMA	F: TCAGGGAGTAATGGTTGGAATG R: GGTGATGATGCCGTGTTCTA
Mmu COL1	F: AGACCTGTGTGTTCCCTACT R: GAATCCATCGGTCATGCTCTC
Mmu fibronectin	F: TACGGAGAGACAGGAGGAAATA R: CATACAGGGTGATGGTGTAGTC
Mmu GAPDH	F: CAAGGTCATCCATGACAACTTTG R: GTCCACCACCCTGTTGCTGTAG
Hsa PTEN	F: CCCACCACAGCTAGAACTTATC R: TCGTCCCTTTCCAGCTTTAC
Hsa PI3K	F: GTCTTGGATGGACTGGCTAAA R: ACAGCTACGATGAGCTTTC
Hsa AKT	F: CTTCTATGGCGCTGAGATTGT R: GCCCGAAGTCTGTGATCTTAAT
Hsa *α*-SMA	F: GAGGTATCCTGACCCTGAAGTA R: AAGCTCGTTGTAGAAGGTGTG
Hsa COL1	F: CTAAAGGCGAACCTGGTGAT R: TCCAGGAGCACCAACATTAC
Hsa fibronectin	F: CTGAGACCACCATCACCATTAG R: GATGGTTCTCTGGATTGGAGTC
Hsa GAPDH	F: ACAACTTTGGTATCGTGGAAGG R: GCCATCACGCCACAGTTTC

## Data Availability

The data are included in this article. If you have any requests, that data will be shared.
